The article "Simulation of Mechanical Heart Valve Dysfunction and the Non-Newtonian Blood Model Approach" was retracted in 2023. Reasons: signs of a paper mill; compromised peer review; unreliable results or conclusions.

# Simulation of Mechanical Heart Valve Dysfunction and the Non-Newtonian Blood Model Approach

**DOI:** 10.1155/2022/9612296

**Published:** 2022-04-19

**Authors:** Aolin Chen, Adi Azriff Bin Basri, Norzian Bin Ismail, Masaaki Tamagawa, Di Zhu, Kamarul Arifin Ahmad

**Affiliations:** ^1^Faculty of Engineering, Universiti Putra Malaysia, Serdang, Selangor 43400, Malaysia; ^2^Faculty of Medicine and Health Sciences, Universiti Putra Malaysia, Serdang, Selangor 43400, Malaysia; ^3^Graduate School of Life Science and Systems Engineering, Kyushu Institute of Technology, Kitakyushu, Fukuoka 804-8550, Japan

## Abstract

The mechanical heart valve (MHV) is commonly used for the treatment of cardiovascular diseases. Nonphysiological hemodynamic in the MHV may cause hemolysis, platelet activation, and an increased risk of thromboembolism. Thromboembolism may cause severe complications and valve dysfunction. This paper thoroughly reviewed the simulation of physical quantities (velocity distribution, vortex formation, and shear stress) in healthy and dysfunctional MHV and reviewed the non-Newtonian blood flow characteristics in MHV. In the MHV numerical study, the dysfunction will affect the simulation results, increase the pressure gradient and shear stress, and change the blood flow patterns, increasing the risks of hemolysis and platelet activation. The blood flow passes downstream and has obvious recirculation and stagnation region with the increased dysfunction severity. Due to the complex structure of the MHV, the non-Newtonian shear-thinning viscosity blood characteristics become apparent in MHV simulations. The comparative study between Newtonian and non-Newtonian always shows the difference. The shear-thinning blood viscosity model is the basics to build the blood, also the blood exhibiting viscoelastic properties. More details are needed to establish a complete and more realistic simulation.

## 1. Introduction

Cardiovascular disease is one of the leading causes of death in the world [1]. Heart valve disease is one kind of cardiovascular disease, and more than 300,000 heart valves are implanted every year worldwide [2, 3]. More than half of them are mechanical heart valves (MHV). Considering its durability and ideal hemodynamic properties, MHV is currently the most common safety choice [4, 5]. However, nonphysiological hemodynamic in MHVs may cause hemolysis, platelet activation, and increased thromboembolism risks [6–12].

The previous numerical studies of MHV mainly concentrated on healthy valves with velocity fields, transvalvular pressure drop, blood component damage, and the downstream flow of normal MHV. The studies also attempted to quantify the relationship between hemodynamics and the possibility of thromboembolic complications [13]. The studies were under steady-state flow conditions [14] and pulsatile flow with or without fluid-structure interaction (FSI) [15–17]. In most studies that considered FSI, the flow through the MHV was laminar [18–20]. Also, direct numerical simulation (DNS) with FSI was performed by Dasi et al. and Nobili et al. [21, 22].

The article "Simulation of Mechanical Heart Valve Dysfunction and the Non-Newtonian Blood Model Approach" was retracted in 2023. Reasons: signs of a paper mill; compromised peer review; unreliable results or conclusions.

Nonphysiological blood flow of mechanical valves leads to being patients at risk of complications of thromboembolism. One of the potential complications associated with mechanical valves is valve dysfunction, which is the dysfunction caused by the formation of pannus and blood clots around the valve structure. It impedes the rotation of one or two leaflets in the BMHV [23]. The frequency of MHV dysfunction is about 0.2% to 6% per year [24]. Smadi et al. [2] performed several different percentage valve dysfunction numerical studies under steady flow. This simulation is the first numerical study dealing with MHV dysfunction to find a noninvasive parameter for dysfunction diagnosis. In vitro, Baumgartner et al. [23] studied the flow through a defective MHV, the result showed that the energy losses decrease with the dysfunction percentage increase, this will noticeably affect the pressure drop at downstream of valve area, and the clear definition between normal and abnormal flows will be difficult.

In the previous study, many researchers have assumed blood as an incompressible Newtonian fluid. This assumption is considered valid as the blood behaves as a Newtonian fluid in large arteries [2, 3, 25], the blood can be assumed as Newtonian [26], leading to some studies assuming blood as a Newtonian fluid when simulating flow through an aorta by the implanted MHV [2, 3, 25, 27, 28]. However, the blood non-Newtonian characteristics may become significant when it passes through the hinge regions of the MHV and the gaps between two leaflets. They can have a significant impact on the wall shear stresses [29]. Alemu and Bluestein [17] simulated blood as a non-Newtonian multiphase fluid and fixed the leaflets to remain fully open. Hanafizadeh et al. [30] simulated blood as non-Newtonian at the diastolic phase of the cardiac cycle. Moradicheghamahi et al. [31] used a fixed grid method to simulate non-Newtonian blood flow passing through an MHV placed in the aortic position.

Sotiropoulos and Borazjani [32] reviewed recent advances and developed a predictive fluid-structure interaction (FSI) algorithm that could simulate BMHV flow with sufficient fine-grained physiological conditions and resolution to explore the link between hemodynamics and blood cell damage. In their review, Zakaria et al. [33] carried out an MHV simulation to study blood clotting potential. The result shows that the vortex formation, recirculation region, and stagnant flow increase the shear stress and residence time in the MHV region, thereby leading to blood clotting. However, in recent years, several authors performed numerical studies on MHV dysfunction [2, 3, 7, 25, 34–37], and the simulation results show a significant difference from the normal MHV. The non-Newtonian viscosity model plays a role in numerical studies of blood flow through the MHV due to the complex structure of MHV [29–31, 36, 38–41].

The article "Simulation of Mechanical Heart Valve Dysfunction and the Non-Newtonian Blood Model Approach" was retracted in 2023. Reasons: signs of a paper mill; compromised peer review; unreliable results or conclusions.

This paper addresses an additional scope for numerical studies of the MHV dysfunction and a non-Newtonian blood flow model for MHV simulation. The review of MHV dysfunction mainly focuses on the one leaflet blocked by the clot and reviews the blood flow patterns in that leaflet dysfunction conditions. The non-Newtonian blood flow part will review the non-Newtonian viscosity blood simulated in MHV, and the different shear-thinning non-Newtonian viscosity blood constitutive model also reviewed some basics of the viscoelastic constitutive model. Finally, conclude the current non-Newtonian blood flow simulation issues in MHV (both normal and dysfunctional conditions).

## 2. Dysfunction Model and Method

Figure 1 shows a typical computational domain used for MHV numerical study [36]. The domain is usually separated into four regions: the upstream region, MHV, aortic root sinuses, and the downstream region. The bileaflet mechanical valve was modeled based on a 25 mm St. Jude Medical bileaflet aortic heart valve [42–46]. There are also nonsymmetric sinuses that were modeled [25, 27, 28, 34–37, 47] based on the in vivo study performed by Reul et al. [48] and used in vitro by Grigioni et al. [49]. Studies by Reul et al. [48] modeled several different valve types and provided relevant primary geometrical data of aortic heart valve prostheses. The simulation investigated flow fields at different types of valves and the mutual interactions between valve geometries. The investigation may eventually lead to the selection of valve types depending on the aortic root geometry. The appropriate adjustment of prostheses could reduce the risk of thromboembolic complications. Choi et al. [28] studied the influence of the aortic root sinus dimensions on the abnormal flow fields in the flow-through MHV. The result indicates that the MHV will lead to high turbulent intensity in the downstream region of the valve and vortex formation in the sinus region. So, if the implant of the MHV is without considering the aortic root geometry, it may produce undesirable hemodynamics, which might result in an increased risk of blood damage and platelet activation.

The article "Simulation of Mechanical Heart Valve Dysfunction and the Non-Newtonian Blood Model Approach" was retracted in 2023. Reasons: signs of a paper mill; compromised peer review; unreliable results or conclusions.

Smadi et al. and Kondo et al. [25, 27] and Emery et al. and Khalili [3, 36] created five defective mechanical valve models. Depending on the opened angles, the dysfunction leaflets are defined as 0% dysfunction (fully opened position) and 25%, 50%, 75%, and 100% dysfunction (fully closed position). Smadi et al. [34] created a pulsatile inlet flow under a two-dimensional dysfunctional MHV model and simulated different dysfunction MHVs in one leaflet. Choi et al. [28] fixed the bottom leaflet in the closed position; the leaflet dysfunction is usually due to the blood clotting at the valve hinge region which could block the motion of leaflets.

The severity of the dysfunction will influence the flow field pattern through MHV [25]. The abnormal increase of blood flow velocity and shear stress, and large vortices also showed vital recirculation around the fixed leaflet [2, 35]. The local velocities, separation regions, and wall shear stress also increase due to leaflet dysfunction [36]. The malfunction also caused higher stresses to develop around the hinges [3]. These stress values exceeded the thresholds corresponding to the elevated risk of hemolysis and platelet activation [37].

For the boundary conditions, Smadi et al. [25] simulated several specific systolic flow rates. However, the rest of the simulations were performed with an experimental pulsatile flow as inlet condition and cardiac output as outlet condition [27, 28, 30, 34–36, 47].  Table 1 describes the dysfunction MHV model, viscosity model, and boundary conditions.

For the MHV dysfunction numerical method, Smadi et al. [25] set the Reynolds number range from 2038 to 5708 based on the inlet boundary condition. This range of Reynolds number agrees with the valve downstream flow turbulent nature [14, 15]. Since the blood flow was assumed to be steady, the Newtonian and turbulent models select standard *k*-*ω* model which was used with 5% turbulent intensity [50, 51]. Smadi et al. [34] introduced the first mesh-free particle method used to study the blood flow through the MHV, demonstrating the SPH method's potential to simulate the complex flow through the MHV. In this study, the shear stress loading on particles was computed based on the concept proposed by Peterson et al. [52]. Yun et al. and Khalili [35, 36] performed a pulsatile inlet flow through MHV during one cardiac cycle. In this study, the blood was assumed as both Newtonian (constant viscosity as 0.0035 kg/(m/s)) and non-Newtonian (the generalized Carreau-Yasuda model), and the standard Reynolds *k*-*ω* turbulence model [53, 54] was also used, which is known to perform well for internal flows. The other dysfunction MHV simulation objectives and results are shown in Table 2.

The article "Simulation of Mechanical Heart Valve Dysfunction and the Non-Newtonian Blood Model Approach" was retracted in 2023. Reasons: signs of a paper mill; compromised peer review; unreliable results or conclusions.

## 3. Simulation of Physical Quantity Dysfunction

### 3.1. Velocity Distribution

Due to the different opening angles of the dysfunction leaflets, the flow fields in the upstream and downstream of the dysfunction MHV were different from the normal MHV, especially the flow separation and vortex formed more obvious in dysfunction MHV [55].

When the percentage of dysfunction increased, shown in Figure 2, the valve becomes more vortical downstream of the MHV, and the number of different scale vortices also has a significant increase. Moreover, a recirculation zone is generated behind the dysfunction valve, especially when the valve is 100% dysfunctional [25].

Smadi et al. [34] used the SPH method in MHV dysfunction simulation during the systolic deceleration phase plotted. The axial velocity of the SPH particles passing at the leading edge and trailing edge of the MHV's leaflets was studied. The results have a good agreement with Bluestein et al. [53], which used the finite volume method and the *k*-*ω* turbulent model. The SPH method simulation results show the consequence of one dysfunctional valve leaflet on velocity, corresponding to a 76% severity in leaflet dysfunction, which leads to a significant increase in the maximal velocity reaching up to 3.52 m/s. Furthermore, the maximal velocity is not located through the central orifice anymore, as expected in the healthy case, but through the lateral normally functioning orifice shown in Figure 3. Under such conditions, the velocity recorded will be 2.2 m/s instead of 3.52 m/s, representing an underestimation of the maximal velocity by 60%. These values agree with the experimental study of Baumgartner et al. [23] and the numerical simulations of Kondo et al. [27].

### 3.2. Vortex Formation

Earlier studies on the flow characteristics of MHV showed that the three orifices of the valve characterized the flow, formed between the sinus and the aortic wall, and formed in the sinus vortex [56–58]. In the MHV model, the upper and lower wall shear layers roll up in the sinus area and form eddies. A single vortex is formed at the peak of the contraction period, and a unique vortex structure still exists early in the deceleration phase. In contrast, in the middle stage of the deceleration phase, the single vortex and other small-scale vortices decompose into two important vortices.

Conversely, periodic vortex shedding was observed after the valve leaflets [15, 27]. Some studies [21, 59] have shown that a shear and flow separation are found downstream of the valve shell and leaflet tips. There are three Valsalva sinuses in the root of the aorta, which makes the area immediately downstream of the aortic valve asymmetrical and significantly impacts the flow domain. When placing the MHV in the aortic position, the geometry becomes more complicated as the valve leaflets expand downstream of the aortic sinus root, which generates a three-dimensional vortical structure and a dynamical recirculation flow within the sinus area [21, 26]. Then, the vortex ring flows into the sinus.

The article "Simulation of Mechanical Heart Valve Dysfunction and the Non-Newtonian Blood Model Approach" was retracted in 2023. Reasons: signs of a paper mill; compromised peer review; unreliable results or conclusions.

Flow disturbance in MHV induces blood constituent activation and damage. Vortex shedding is due to the vortices' complex flow [60]. Vortex shedding was postulated in flow-through MHV [61] and observed experimentally [53, 62]. When the blood flows through the mechanical heart valve generates a shear layer, this layer is prone to vortex shedding due to an invisible instability. When the blood flow accelerates and passes the MHV orifice, the eddy ring will periodically roll into a vortex column and tear from the edge.

Further downstream, the vortex becomes turbulent [63, 64]. Vortices of different length scales mainly characterize the turbulent flow. When the vortex length matches blood components' size, it will lead to blood damage (hemolysis) and thrombus formation (platelet activation). Most experimental and numerical studies on MHV showed many times high of turbulent and wall shear stress around the leaflet than the physiological ones [13, 15, 16], potentially leading to blood component damage.

Huang et al. [65] performed the first high-resolution unsteady laminar flow numerical simulation in a tilting disk heart valve. The complex behavior of vortex shedding found an optimal environment for activated platelets and clotting factors. The platelet activation level is calculated numerically by the sum of the shear stress intensity at each instant on different paths multiplied by the residence time. Under the turbulent conditions, the particle paths were calculated based on the stochastic model [66]. Bluestein et al. [53] have used and described in detail this model.

When the percentage of dysfunction increased MHV, the downstream flow fields became more vortical [25]. In a partially defective leaflet (50%), the flow behavior has changed dramatically. The vortices are generated between two leaflets and the sinus area during the acceleration stage. Compared with the normal MHV, dysfunction MHV-formed vortices appeared earlier during the systolic phase. Compared with normal cases, defective leaflets are more prone to vortex shedding behind the valve. There has a significant difference between the case of 100% dysfunction MHV and partial dysfunction at upstream formed by a vortex structure, just before the leaflet is completely closed. Moreover, a recirculation region was formed behind the dysfunction leaflet, especially in the complete dysfunction case [27].

The article "Simulation of Mechanical Heart Valve Dysfunction and the Non-Newtonian Blood Model Approach" was retracted in 2023. Reasons: signs of a paper mill; compromised peer review; unreliable results or conclusions.

With the number and scale increased of vortices, the valve's blood residence time downstream will increase. As a result, this will increase the level of platelet activation and thrombosis. Studies have shown that in moderate levels of dysfunction, platelet activation is significantly increased, which may cause thrombosis or worsen thrombosis. Also, leading to a vicious cycle, the abnormal flow fields accelerate the thrombosis formation on the valves, which aggravates valve dysfunction, which is shown in Figure 4. However, in the case of complete dysfunction, the downstream occurred low levels of vorticity due to the block of dysfunctional leaflet formed by a low-velocity region [35].

### 3.3. Shear Stress

When the blood flow passes through the MHV, it will generate a high-pressure drop, resulting in recirculation and stagnation [67–70]. The increase of shear stress will lead to blood damage (hemolysis) and platelet activation. The change of flow pattern causes platelet aggregation [71, 72].

Turbulent shear stress (TSS) is generated by valve-induced turbulence, which is usually focused on studying blood hemolysis [13]. Many studies have characterized shear stress and RSS in MHV [13, 26, 73, 74]. Yin et al. and Morshed et al. [75] reviewed the dynamics in MHV and explained how the TSS could contribute to hemolysis and platelet.

Wall shear stress refers to the force per unit area exerted by the wall on the fluid in the direction of the local tangent plane [10]. When the blood flows through the MHV, the red blood cell can be damaged by shear stress on the order of 1 to 10 [76]. When exposure time is within physiological ranges, shear stresses can happen platelet activation on the order of 20 to 60 [76]. The shear stress is not the only determining factor causing the hemolysis and the activation of platelets. The exposure time is another critical factor [77]. The hemolysis can occur at the TSS in the range of 400-5000 within an exposure time of 10 ms [3, 78]. The platelet activation and hemolysis will increase the risk of blood clot formation [20]. The clot may detach and block the arteries, leading to embolism and stroke [79, 80].

Several studies [81–83] suggested that the shear stress is highest in the hinge regions and with obvious reverse flow and stagnation. When the flow passes through the hinge region, it will generate high shear stress, which is the main factor cause of platelet activation [20, 67, 84, 85]. In MHV, the hinge gap width's geometry has a significant impact on the leakage flow structure and markers of platelet damage [77, 85–87]. When passing through the hinge area, the clot may deposit in the hinge and form a thrombus, which is detrimental to the function of the valve.

The article "Simulation of Mechanical Heart Valve Dysfunction and the Non-Newtonian Blood Model Approach" was retracted in 2023. Reasons: signs of a paper mill; compromised peer review; unreliable results or conclusions.

In dysfunction MHV, with the percentage of dysfunction increased, the TSS level and highest value position will change; the TSS-affected regions move to the upper side of the valve [50]. The number of blood elements exposed to a high shear stress area will increase, and more vortices also increase the resident time, which will significantly increase the level of platelet activation and thrombus formation; the dysfunction valve caused abnormal flow could lead to a vicious cycle.

From the physical quantity review of the dysfunction MHV, it is obvious that the dysfunction changed the blood flow patterns in MHV, increased the maximum velocity and shear stress, and increased the number and scales of vortices. Those results will lead to hemolysis and thrombosis formation or worsen thrombosis, which will also induce a vicious circle. Obvious recirculation and stagnation region will decrease the shear stress, and downstream of complete dysfunction occurred in low-velocity region that is meaningful to assimilate the blood flow as a non-Newtonian flow.

## 4. Non-Newtonian Blood Flow

### 4.1. Non-Newtonian Blood Flow Simulation

Blood is a complex fluid consisting of blood cells suspended in plasma. The shear-thinning behavior depends on the properties of the suspended particles [88]; the blood viscosity is the relationship between shear rate and hematocrit [89]. Due to the larger shear rates experienced by blood cells in the larger vessels, the effective viscosity becomes asymptotically constant, and the blood could be assumed to behave as a Newtonian fluid [90–94]. The Newtonian blood viscosity assumption simulation is a valid approach because the simulation result did not have a significant difference between the Newtonian and non-Newtonian viscosity models [95].

Several factors can affect blood viscosity, like hematocrit, plasma viscosity, vascular diameter, and temperature [96–98]. The non-Newtonian viscosity behavior is mainly affected by the aggregation of red blood cells and the rouleaux, especially in low shear rates [99]; the shear forces break up the rouleaux into small stacks, and the dissipation is dependent on the rate of shear [100]; when the dissipation increases, the viscosity will decrease, a condition known as a shear-thinning behavior. Several studies with human blood [101, 102] have shown the variation of the effective viscosity with the shear rate. The rate of strain is about (depending on the hematocrit level) in vivo vessels, the non-Newtonian viscosity behavior becomes less important, and the effective viscosity approaches an asymptotic value.

The article "Simulation of Mechanical Heart Valve Dysfunction and the Non-Newtonian Blood Model Approach" was retracted in 2023. Reasons: signs of a paper mill; compromised peer review; unreliable results or conclusions.

In reality, the blood flow in the aorta is pulsatile and transitional. The flow is very inhomogeneous, which means the previous assumption might be incorrect. The Newtonian model is not suitable for all situations. The transient shear rate over one cardiac period in the aorta [102]. In a cardiac cycle of the pulsatile flow, most of the mean flow rate is zero, so the shear rate is low. Even at a high flow rate region, it will generate recirculation and resident region. Experimental studies [103, 104] have shown that the blood behaves non-Newtonian in pulsatile flow and when the shear stress less than the blood exhibits shear-thinning properties, which is one significant characteristic of non-Newtonian blood [102]. When the characteristic length becomes comparable with the size of red blood cells, the blood flow can also be considered non-Newtonian flow. Consequently, in the MHV model, the microflow in the complex structure of leaflet gaps and hinge region would contain a broad range, and the sizes of microstructure are comparable with red blood cells. Therefore, non-Newtonian blood viscosity characteristics are significant in the numerical simulation study of MHV, yielding more realistic results.

### 4.2. Shear-Thinning Non-Newtonian Blood Flow in MHV

Viscosity plays a vital role in induced shear stresses. Various models have proposed [105] to describe the shear-thinning and viscoelastic properties of the blood [106, 107]. In the case of MHV exit a wide range of shear stress, the non-Newtonian viscosity exhibits a more important effect. The exact viscosity model is necessary to get the accurate viscosity effect. Many non-Newtonian mathematical models are created to describe shear-thinning blood viscosity [108, 109]. The Carreau [30, 40, 110] and Carreau-Yasuda [111, 112] models are most frequently used in the literature.

The Carreau-Yasuda constitutive model was most commonly used to describe non-Newtonian blood due to its reported property of viscosity changes that are more accurate [30, 31, 113, 114]. Hanafizadeh et al. [30] and Moradicheghamahi et al. [31] have recommended this model used in the numerical simulation of non-Newtonian blood flow in the MHV model. Moradicheghamahi et al. [31] performed a numerical simulation in MHV and used the Carreau-Yasuda model to describe the non-Newtonian blood. The result shows that the prediction of hemolysis is dependent on the fluid model. Choi and Kim [115] built the blood flow of a Newtonian and non-Newtonian flow with the Carreau model, and the result shows that leaflet motions and blood flow are similar for the Newtonian and non-Newtonian cases, but the non-Newtonian case generates higher shear stress. Abbas et al. [41] also used the Carreau-Yasuda model to describe the non-Newtonian blood flow in MHV and study the platelet activation potential. The numerical result has good agreement with experimental measurements by Yin et al. [116]. When considering the specific patients, the blood non-Newtonian characteristics can be affected by the temperature and blood oxygen concentration directly. The Carreau model is not easily adapted due to the lack of parameters connecting the clinical counterparts. The Quemada model [117] has additional parameters for determining blood behavior using blood cell-specific volume. Marcinkowska-Gapińska et al. fit their data to the three non-Newtonian models (Casson, Ree-Eyring, and Quemada) and concluded that the Quemada model was the most suitable [118].

The article "Simulation of Mechanical Heart Valve Dysfunction and the Non-Newtonian Blood Model Approach" was retracted in 2023. Reasons: signs of a paper mill; compromised peer review; unreliable results or conclusions.

In the study of the difference between the non-Newtonian and Newtonian models, the Newtonian model generates lower wall shear stress. In the non-Newtonian model, the Cross model shows a significant difference [119]. Doost et al. conducted a simulation of blood flow using patient-specific geometry with several viscosity models, including the Newtonian, Carreau, Casson Cross, Power Law, and K-L model. They conclude that the non-Newtonian models would significantly affect the numerical simulation result [110].

The MHV is an unnatural structure, and small gaps will be formed when it is at its closing position and around its hinges. There are small regions of different flow domains at valve hinges. In the numerical simulation of flow patterns in the hinge regions, the micro size of the hinge gaps should be taken into account. When the physical size is comparable with the characteristic length of red blood cells, the non-Newtonian viscosity blood assumption is important [59], especially [27, 59]. In the leaflet gaps and hinge regions that contain a broad range of shear stress, considering the shear stress acting on blood elements, the non-Newtonian blood will yield a more realistic result [30]. Many MHV simulations are simplified with the MHV structure without details of the hinge region to accelerate the simulation speed. The real structure is complex; the stress should be higher and consequently more dangerous for hemolysis [120].

### 4.3. Shear-Thinning Non-Newtonian Viscosity Models

There are more than eleven kinds of the non-Newtonian models (Casson, K-L, Modified Casson, Carreau, Carreau-Yasuda, Cross, Power Law, Modified Power Law, Generalized Power Law, Ree-Eyring, and Quemada) applied to define the rheology of blood flow. All of these non-Newtonian shear-thinning viscosity models are the most famous models that can simulate non-Newtonian blood flow.

The article "Simulation of Mechanical Heart Valve Dysfunction and the Non-Newtonian Blood Model Approach" was retracted in 2023. Reasons: signs of a paper mill; compromised peer review; unreliable results or conclusions.

The simplest type of model to account for shear rate-dependent viscosity is the Power Law model. This model has two parameters: the *k* and *n* (dimensionless) are selected to fit experimental data. When *n* = 1 and *k* = *μ*, the model reduces to the Newtonian case. For *n* > 1, the model represents shear thickening, whereas for *n* < 1, it represents shear thinning [121]. The limitation of the Power Law model is that it cannot describe the viscosity at small shear stress. The Modified Power Law and Generalized Power Law models are built to improve the scope of application [108, 122].

The viscosity model has two main types. The first is the shear-dependent type, which equation can be written in the general form.

Different choices of the function correspond to different blood flow models. The model parameters are easily affected by many factors like hematocrit, temperature, plasma viscosity, age of RBCs, and exercise level or gender. The Cross, Carreau, and Carreau-Yasuda models include this type.

Another type is the yield stress type. When the shear stress is less than the yield stress, the fluid exhibits a solid-like behavior. Thus, the fluid flows depending on the yield stress and requires a minimum pressure gradient to drive the fluid. Casson's constitutive equation is the typical yield stress type non-Newtonian viscosity model, which has zero viscosity at an infinite rate of shear and infinite viscosity at zero rates of shear [123]. The Quemada model also is a yield stress type, which included concentration ratio in his model, which will be interpreted as hematocrit here. The Quemada model can be used in specific patient numerical studies in different hematocrit conditions [39].

### 4.4. Non-Newtonian Viscoelastic Model

Whole blood is a concentrated suspension of formed cellular elements, which exhibits non-Newtonian characteristics due to the erythrocyte aggregation at low shear rates. Except for shear thinning, viscoelastic and thixotropic are also important non-Newtonian behaviors of the blood [124].

Blood cells are essentially elastic membranes filled with fluid; RBCs can form aggregates, called rouleaux, at low shear rates; the rouleaux aggregates and stores elastic energy, with the fluid flow; the sliding of internal cellular needs input energy; this energy dissipated through friction and later gradually disaggregated into cells at high shear rates [125]. Elastic energy exhibits stress relaxation and the bridging mechanism within the structure. The relaxation time depends on the shear rate. With a shear rate of the order of 10 s^−1^, the elastic nature of the blood is negligible, as evidenced by the combination of oscillation and stable flow viscosity. However, in the circulatory system, use the viscoelastic constitutive equation to model the blood; the finite viscoelastic behavior of the blood should be taken into account. Blood viscoelasticity also is dependent on factors such as temperature, hematocrit, and RBC characteristics [7].

The article "Simulation of Mechanical Heart Valve Dysfunction and the Non-Newtonian Blood Model Approach" was retracted in 2023. Reasons: signs of a paper mill; compromised peer review; unreliable results or conclusions.

There are several different kinds of viscoelastic models used to describe the viscoelastic blood fluid dynamics. There are three types of governing equation building viscoelastic extra stress: statistical models, integral models, and differential models. In which the differential models describe the viscoelastic extra stress tensor by a partial differential equation, it was widely used in numerical simulation due to its easy implementation in current CFD codes; the Johnson-Segalman differential viscoelastic constitutive model is widely used in a blood flow numerical study [126]. The well-known Maxwell and Oldroyd-B models are the special cases of the Johnson-Segalman models.

Recently, the generalized Maxwell model [127, 128] and generalized Oldroyd-B model [129, 130] have been proposed and improved. These models have been successfully extended to 3D simulations [130, 131] and have good agreement with experimental data.

Higher shear rate is generated in the large arteries, the blood flow can be assumed as Newtonian flow in many review studies [132]. Although the shear rate is generally high in large arteries, some cardiovascular disease induces blood flow disturbance and generates stagnant and recirculation regions, significantly reducing the shear rate [133]. When the blood flows through the MHV, the recirculation, stagnation, vortex structures, and flow separation are obvious, which enhance the probability of occurrence of low shear rates and require the use of the non-Newtonian models [21, 26, 35, 67–70]. In dysfunction MHV simulation, the blood flow behind the dysfunction leaflet has more significant recirculation flow and stagnation. Several studies have studied the shear-thinning non-Newtonian viscosity models in MHV [17, 30, 31]. However, none of them consider the viscoelastic properties of the blood.

The shear-thinning non-Newtonian viscosity model has been used in many MHV numerical studies, except for shear thinning. Also, viscoelastic is an important non-Newtonian behavior of the blood; the generalized Holroyd-B model can build shear-thinning and viscoelastic characteristics, has successfully extended to simple 3D simulation, and it is still full of challenges for complex 3D structures like MHV.

The article "Simulation of Mechanical Heart Valve Dysfunction and the Non-Newtonian Blood Model Approach" was retracted in 2023. Reasons: signs of a paper mill; compromised peer review; unreliable results or conclusions.

## 5. Issues and Recommendations

The human aortic wall is compliant; the compliance of the aorta determines its increase in pressure [105, 134]. A rigid wall will generate higher pressure variations, and the blood will exhibit non-Newtonian properties in the low-velocity regions. If the arterial walls are assumed as rigid, this neglects the contact mechanics in the valve region in the low-velocity flow regions. The elastic wall may lead to a reduction in the reaction forces and wall shear stresses [30].

Studies with a flexible aortic root can be performed to recapitulate better physiological conditions in the FSI model [135]. The explicit coupling method works well with the mechanical valve simulation with rigid leaflets. The difference between weak and strong coupling is in their ability to promote numerical stability, and both methods are numerically accurate. A simulation employing strong coupling will be necessary for the simulation to be extended to the MHV to accurately simulate the complex 3D motion of the leaflets during a cardiac cycle [19].

Additionally, the simplification of hinge structural integrity in BMHVs and without applied friction will affect the microflow near the leaflet hinges. Hinges with a wide gap (around) [136] lead to non-Newtonian behavior under specific conditions [27, 59]. Non-Newtonian effects near the hinge region are significant. The magnitude of the shear stress error predicted will be up to 80% if the blood is assumed to be a Newtonian fluid [30]. The hinge geometry is modeled by simplification, and it is plausible that the stress in a real valve would be even higher [59].

Results are always different in comparative MHV numerical studies between Newtonian and non-Newtonian fluids because there has much difference in the parameters for the non-Newtonian viscosity model and even for the structure of the model itself [40]. The shear-thinning non-Newtonian viscosity model is the first step toward the realistic simulation since the blood also exhibits viscoelastic properties; the model should account for the time history of the rate of strain. Also, the viscoelastic model has not yet been implanted into a numerical simulation of MHV. In previous non-Newtonian numerical studies, only the Carreau-Yasuda [27, 29–31, 36, 38, 40, 41] and Quemada [39] viscosity models were used in MHV simulations. Many studies had compared different non-Newtonian viscosity models in carotid bifurcations [31, 47, 137, 138], aortic arch [119, 139], and arteries with consecutive stenosis [140, 141]. The different non-Newtonian models show a difference in axial velocity values [140] and WSS [116, 119, 137]. In MHV numerical studies, the different non-Newtonian model comparative studies should be meaningful.

The article "Simulation of Mechanical Heart Valve Dysfunction and the Non-Newtonian Blood Model Approach" was retracted in 2023. Reasons: signs of a paper mill; compromised peer review; unreliable results or conclusions.

## 6. Conclusions

The current review compiled studies carried out on the dysfunctional MHVs and non-Newtonian models of MHV. In the dysfunction condition, the dysfunction model is usually with one healthy leaflet and one dysfunctional leaflet with several different percentages of dysfunction. The results show that the maximum blood velocity increased with the effective orifice area decrease. Dysfunctionality increases the transvalvular pressure gradient, flow separation, growing eddies, stagnation, and recirculation. Heart valves induce flow disturbances that play a role in blood constituent activation. When the percentage of dysfunction security increased, there has a significant increase in the number of vortices and creates conditions for thrombus formation, which will worsen the valve dysfunction.

Blood is a complex fluid composed of blood cells suspended in plasma. Due to the presence of these particles, the blood exhibits a non-Newtonian behavior, and its viscosity is vital in the shear stress of the walls and particles. Non-Newtonian characteristics include shear-thinning and viscoelastic behavior. The shear-thinning viscosity models are widely used in MHV blood flow simulation. In the hinge recesses of MHV and the gap between two leaflets during a leakage phase, the non-Newtonian effect of the blood may become apparent. In order to build an accurate blood model, changes in blood viscosity must accurately be observed, and the Carreau-Yasuda viscosity model is most commonly used in shear-thinning non-Newtonian MHV blood flow simulations. However, the viscoelastic model still not be used in the previous study. Some studies also found that simulations of Newtonian fluids and non-Newtonian or between different non-Newtonian models will yield different results, such as higher shear stresses for non-Newtonian fluids. Although the current results are still different, creating more models to simulate and compare conditions will help solve the problem and allow for better studies of the failure mechanism and preventive measures of MHV dysfunction.

## Figures and Tables

**Figure 1:** BMHV structure and computational domain [36].

**Figure 2:** Coherent structure downstream of a normal and a defective mechanical valve for 7 L/min [25].

**Figure 3:** Flow patterns through a dysfunctional BMHV at peak systolic (0.1 s) and early deceleration phase (0.3 s): (a) velocity magnitude, (b) vorticity, and (c) turbulent shear stress [6].

**Figure 4:** Vorticity distributions and coherent structure downstream of a healthy and a dysfunctional mechanical valve at different time instants [34].

The article "Simulation of Mechanical Heart Valve Dysfunction and the Non-Newtonian Blood Model Approach" was retracted in 2023. Reasons: signs of a paper mill; compromised peer review; unreliable results or conclusions.

**Table 1:** Comparison of the MHV dysfunction model.

Author	MHV model	Viscosity model	Inlet condition	Outlet condition
Smadi et al. [25]	25 mm St. Jude Medical hemodynamic plus valve	Newtonian	7.5, 10.5, 15, 18, and 21 L/min	2.5, 3.5, 5, 6, and 7 L/min
Smadi et al. [2]	25 mm St. Jude Medical hemodynamic plus valve	Newtonian	Pulsatile	5 L/min
Smadi et al. [34]	25 mm St. Jude Medical hemodynamic plus valve	Newtonian	Pulsatile	5 L/min
Bessonov et al. [7]	St. Jude Medical bileaflet aortic heart valve	Newtonian	Pulsatile	5.5 L/min
Yun et al. [35]	St. Jude Medical (SJM) valve	Newtonian and non-Newtonian	Pulsatile	\
Emery et al. [3]	25 mm St. Jude Medical hemodynamic plus valve	Newtonian and non-Newtonian	Pulsatile	5 L/min
Khalili [36]	25 mm St. Jude Medical hemodynamic plus valve	Newtonian	Pulsatile	5 L/min

**Table 2:** MHV dysfunction simulation objectives and results.

Author	Dysfunction position	Objectives	Result
Smadi et al. [25]	0%, 25%, 50%, 75%, 100%	Develop parameters used for early noninvasive diagnosis of such valve malfunction.	The flow of the defective valve is highly influenced by the malfunction severity. Proposes to test two potential noninvasive parameters.
Smadi et al. [2]	0%, 25%, 50%, 75%, 100%	Numerically and experimentally investigate the pulsatile turbulent flow downstream of a dysfunctional bileaflet mechanical heart valve.	The flows downstream of a dysfunctional valve were characterized by abnormally elevated velocities and shear stresses as well as large-scale vortices. The maximal velocity in the lateral orifice could be an indication of valve dysfunction.
Bessonov et al. [7]	From 25% to 100%	SPH applied to study the flow through normal and dysfunctional BMHVs.	The accumulation of shear stress patterns on blood components illustrates the important role played by nonphysiological flow patterns and mainly vortical structures in this issue.
Yun et al. [35]	100%	Numerically study flow dynamics that occur in the vicinity of BMHVs using a fluid-solid coupling method that combines lattice Boltzmann fluid modeling.	In severe dysfunction cases, a strong jet is seen at the top orifice, as well as through the central orifice. The vorticity magnitude is stronger and also shows strong recirculation of flow near the fixed bottom leaflet.
Emery et al. [3]	0%, 25%, 50%, 75%, 100%	Analyse velocity, pressure drop, wall shear stress, and vorticity profiles to better understand the blood flow through the dysfunctional leaflet.	Leaflet dysfunction caused increased local velocities, separation regions, and wall shear stresses. When dysfunction increased, the pressure drops increased. The leaflet dysfunction also caused higher stresses developed around the hinges.
Khalili [36]	0%, 25%, 50%, 75%, 100%	Study the flow characteristics through valves during their normal operation and dysfunction.	Maximum flow velocities and turbulent shear stress increased with increase of dysfunction. These stress values exceeded the thresholds corresponding to the elevated risk of hemolysis and platelet activation. The regions of elevated stresses were concentrated around and downstream of the functional leaflet.

The article "Simulation of Mechanical Heart Valve Dysfunction and the Non-Newtonian Blood Model Approach" was retracted in 2023. Reasons: signs of a paper mill; compromised peer review; unreliable results or conclusions.

## Data Availability

The datasets used in this paper are available from the corresponding author upon request.
